The article "Analysis of the Correlation between College Music Education and Public Mental Health Based on Deep Learning" was retracted in 2023. Reasons: signs of a paper mill; suspected computer-generated content; unreliable results or conclusions; concerns about the data.

# Analysis of the Correlation between College Music Education and Public Mental Health Based on Deep Learning

**DOI:** 10.1155/2022/6593850

**Published:** 2022-10-05

**Authors:** Jingle Huang

**Affiliations:** College of Music and Dance, Zhengzhou Normal University, Zhengzhou 475000, China

## Abstract

With the continuous changes of college music education and public mental health problems, conventional solutions are no longer sufficient. At this time, we adopted a method based on deep learning to study them. The experiments showed that ① deep learning can be well integrated into two. Among them, the rapport rate between them reached 91%, and the sometimes-unstable state of the system was solved by optimizing the model. Finally, through the evaluation algorithm, the overall score of the model was obtained to fluctuate between 85 and 90. ② According to the data in the figures and tables, it can be concluded that university music education under deep learning has received more attention in my country, and the investment amount has also increased from 2.4 billion to 3.7 billion. The highest music education activities in universities have become 55% of concerts and 41% of musical instrument experience classes, and finally, my country's public mental health problem has become a country with the lowest level in the world.

## 1. Introduction

Deep learning can have many computing models to learn abstract data, and many top technologies are applied in it. It uses back propagation algorithm to solve the structural and complex problems of big data, so that the machine itself can change the data to represent each data. Layers, deep convolutional networks, and recurrent networks have all achieved great breakthroughs under the influence of deep learning [1]. Deep learning is applied to artificial neural networks, in which pattern recognition and machine learning have won major competitions. The biggest difference between deep learning and shallow learning is the depth of their credit paths, and they learn through these paths. The causal link between deep, unsupervised learning is widely spread in high-tech [2]. Deep learning algorithms still need to be continuously updated. In the update, great success has been achieved in several fields of vision and language. These algorithms have been able to be trained in deep learning models, but how are they trained without supervision? What goes down? Experimental investigations were conducted to this end, with results showing that unsupervised pretraining steers training to the least attractive regions that support optimal generalization to the training set; evidence from these results supports the interpretation of training [3]. In order to solve the noncoding mutation effect of sequence identification in human genes, a deep learning algorithm framework was developed. This model framework can directly learn the gene sequence code in chromatin, so that the mutation situation can be predicted in advance, and this feature can be used to improve gene: the order of variation [4]. Deep learning is widely used in medicine. It mainly helps some problems in medical images. The depth is constantly improving to improve the functions of many medical machines. The application of deep learning in image anatomy, cell result inspection, and auxiliary diagnosis is reviewed. Basic knowledge provide some directions for future deep learning research [5]. To explore the causal relationship between factors affecting educational satisfaction in order to improve the quality of college music education, and to make recommendations for educational satisfaction by analyzing this causal relationship, the willingness to learn has a positive impact and a negative impact on the learning process, and research shows the need to improve the quality of college music education by creating an educational environment that promotes motivation and immersion in learning, thereby increasing student satisfaction with education [6]. The colonial nature of music education in Nigerian universities is a serious issue, and he uses the framework of polycolonialism to see the Nigerian higher education system as a historical and contemporary relic of colonialism, where Nigerian universities are engaged in the production of musical knowledge. It is based on information from academic sources that must be critiqued, questioned, transformed, revised as needed, and studied in context, context, and comparison, and it has been suggested that decolonization of academic music education in any society implies a focus on creating, understanding, and sharing musical knowledge of diversity and affiliation [7]. College music education is closely related to culture. It is an important cultural heritage carrier of human beings, carrying the essence of human civilization. Our broad and profound national culture is the treasure house of Chinese culture. Education and cultural heritage go hand in hand. University music education is an important means to popularize ethnic music culture, and conservatories are the main link of ethnic music culture. Finally, the importance and role of ethnic music culture in the popularization of music in higher education are proposed, and specific implementation methods and means are proposed [8]. In order to study issues such as university music education, an in-depth look at several university music institutions in France, the UK, Poland, and other European countries, although similar institutions in the former Yugoslav capital deal with the same topics as the Zagreb Academy of Music, here, the other EU countries mentioned have well-organized university-level music institutions, only one, thus becoming one of the most important institutions of the Zagreb Academy of Music [9]. University music education is an important part of quality education in public universities. Based on the current development status of music education in many domestic colleges and universities, the relevant achievements of higher education in my country are sorted out, the shortcomings and roots of music education in colleges and universities are analyzed, and corresponding measures are put forward. The countermeasures and suggestions put forward concrete solutions [10]. Substance nonadherence is a very serious problem in public mental health, and numerous studies have been carried out on it. Using information on patterns, screening programs that identify those most likely to be nonadherent in this population may be more effective [11]. DBT can be well used to treat BPD patients in public mental health, and we propose a long-term experimental comparative study of six months versus only four days of treatment in hospital settings and in public mental health settings. It is a very good approach to provide DBT therapy to patients [12]. There are many models of public mental health services in the United States, and it has been suggested that analyzing the different patterns of inpatient and outpatient mental health service use among Asian Americans may shed light on the reasons for their widespread overuse; in particular, despite many studies showing that Asian Americans tend to underutilize mental health services, this study identifies racial differences between groups and subgroups using inpatient and outpatient mental health services and mental health referral resources and discusses their impact: these findings of clinical and research findings [13]. There is a survey of 50 people in Australia with public mental health problems, their average age is in their 30s, most patients are unmarried and unemployed, schizophrenia is common and expensive to treat, such records can help the healthcare system identify patients in this subgroup and guide management strategies for these often disadvantaged and disadvantaged patients [14]. Public mental health includes promoting mental health, preventing mental disorders and suicide, reducing mental health inequalities, and managing and organizing mental health services. Modern mental health public policy aims to improve mental health by influencing mental health determinants in all areas of public policy. The stigma of mental disorders is a pervasive phenomenon that creates barriers to seeking care and developing health services and has become an important issue in the public health response [15].

## 2. Deep Learning Analysis

### 2.1. Definition of Deep Learning

Most modern deep learning models use neural networks. Cumulative neural networks, although they may consist of propositions or hidden variables, arranged hierarchically in deep genomic models, such as in deep learning. Each level of training changes a certain input type. Aggregate and abstract inputs in image recognition applications, the last one can design the shape of a human face. The caveat is that in deep learning, you will find which level the function is best suited for. The “depth” in “deep learning” refers to the number of levels of data transformation. In particular, the deep learning system is very deep in the credit allocation roadmap (CAP); for this network, the signal can pass through a layer multiple times, and the depth of the CAP can be unlimited. And there is no generally accepted depth threshold that differentiates surface learning from deep learning. Most researchers agree that WTP depth > 2; in deep learning, a CAP depth of 2 is considered a general approximation since it can simulate any function. That is, more layers do not increase the network capacity of WTP. Deep models (CAP > 2) estimate features that can have more features than flat versions. Therefore, additional layers help to study properties. Deep learning architectures are often built using a layered approach, and deep learning can help you understand these abstractions and identify features that can improve efficiency. For supervised learning problems, deep learning works by transforming the data into a compact intermediary representation similar to the parent component and removing redundant representations, which is a significant advantage since unlabeled data contains more information than labeled data. Examples of deep structures that can be trained without supervision include neural history and deep belief networks.

### 2.2. The Difference between Deep Learning and Shallow Learning

Shallow learning is a machine learning method that gets the job done. Students casually accept and please both and get information about scars when it does not matter when they get and get. Such a review results in memorizing exam prep exercises in a short amount of time, which does not help, and facilitates long-term understanding and retention of knowledge and information that students forget immediately after class. Superficial learners need external forces to stimulate learning. Often, grading, passing, and conferring degrees are usually done to facilitate student learning. The purpose of learning is not to fail or fail an exam. Students are only interested in the knowledge content of the next exam. Deep learning means that students can critically learn and incorporate new concepts and facts, into raw mental structures, by making connections between disparate ideas and integrating existing ones, mechanically compared to surface learning and passively acquire knowledge and store data separately. Deep learning emphasizes active and critical learning of learners. The learner must understand the full meaning of the content, including the connections between the content and with other topics and ideas, as seen by the definition of deep learning, which involves critical reflection and avoidance of passive acquisition of knowledge, including integrating what students develop. The information needed is also lifelong learning. In terms of time and space outside the school, after various restrictions, everyone's demand for deep learning will be stronger.

### 2.3. Applications of Deep Learning

Automatic speech recognition is the first and most interesting success case of deep learning, and LSTM neural network can learn tasks. In “extremely deep learning” at intervals of seconds, speech events are separated by thousands of discrete time steps. One of them is about 10 ms. LSTMs with forget filters are comparable to task-based speech recognition. According to TIMIT, the initial success of speech recognition was only a small recognition task. Image recognition is as follows: like TIMIT, its small size allows users to try multiple configurations. There is a list of all the results of this collection, which first appeared in 2011, and the vehicle can perform multifaceted rotation monitoring after adding deep learning. Visual art processing is as follows: increasing the use of deep learning methods in various visual arts, closely related to the advancement of image recognition, the proven DNN function can generate engaging images based on random visual input fields and provide an interesting browsing experience. Natural language processing is as follows: neural networks have been used for language modeling since the early 2000s. LSTMs have helped improve machine translation and language modeling. Other techniques in this area include word sampling and word embedding. This can be seen as a layer of representation in deep learning architectures, representing positions as points in vector space relative to other elements in the dataset. Medical image analysis is as follows: deep learning provides results comparable to other methods. In medical applications such as cancer cell classification, lesion detection, organ segmentation, and image improvement, mobile advertising is as follows: finding the right mobile audience for mobile advertising is always a challenge. This is because many data points need to be validated and processed before an ad server can be created and used. Use audiences to serve ads. Image restoration is as follows: deep learning can solve image problems such as distortion, high resolution, color correction, and film color correction. These applications include training methods such as field reduction for efficient retrieval of training images on image datasets and enhanced depth-of-field reproduction on newly created images.

### 2.4. The Relationship between Deep Learning and the Human Cognitive Domain and Brain

Deep learning is closely related to a class of brain development theories proposed by cognitive neuroscientists in the early 1990s and adopted as computer models. Making them the precursors to deep learning systems, these developmental models are generally characterized by the self-organization of available support in the brain for various learning dynamics. It is like neural networks used in deep learning models, and neocortical neural networks use a hierarchy of filters, where each layer processes data from the previous layer and redirects its output to another layer. This process produces a self-organizing stack of sensors that can easily adapt to the work environment, so-called trophic factor waves, where different regions of the brain connect in tandem, with one layer of tissue maturing before another. Wait until the whole brain is fully grown using various methods. On the other hand, to test the viability of deep learning models from a neuroscience perspective, we identified variables. In the inverse diffusion algorithm, which improves the processing realism, other researchers believed that unsupervised deep learning models such as hierarchical phylogenetic models and deep belief networks can estimate biological reality. In this context, neural network models have been linked to model-driven neural processing data in the cerebral cortex; although, there are no systematic comparisons between the organization of the human brain and deep neural encoding and similar reports, for example, that computations done by deep learning modules can be like real neurons and populations of neurons, and that deep learning models developed perform similarly to real neurons by showing the primate visual system measured at the individual and population levels.

## 3. Research on Public Mental Health Model

① During initialization, *k* sample points are randomly selected from the *N* initial samples and use it as the cluster center. ② Calculate the Euclidean distance from each remaining sample in ① to the cluster center *k* according to formula (1). ③ According to the calculation results in ②, divide each sample into the closest one. ④ Calculate the groups centered on each new group and then use formula (7) to calculate the SSE values for all groups. ⑤ Check whether the total SSE value changes. If there is a change, return to ②, if not ⑥, then ⑥ grouping ends, and the final result of the grouping is displayed.

### 3.1. Create a Database of Public Mental Health Models

The purpose of grouping is to group objects with similar properties. The data collected is unlabeled in most cases, and grouping can separate the data into different groups, the more similar the data within each group. And the data between groups is unique, and most grouping algorithms belong to partition-based grouping, density-based clustering from tables, density-based clustering, and instance clustering that are one of the most common techniques in traditional machine learning algorithms. Cluster analysis is popular for its usefulness, simple, and efficient. It has been successfully used in many fields such as document synthesis. In this study, we chose a *K*-means clustering algorithm to separate the number of meals and entropy of students. The algorithm is a partition-based grouping algorithm. It has the advantages of good efficiency, easy to understand, and fast calculation speed. The main idea of the *K*-mean clustering algorithm is as follows: first, a database is designed, *k* sample points are randomly selected from a database and take it as the center of the cluster, and the calculation formula is

(1) $$\begin{array}{c} d\left(x,C_{i}\right)=\sqrt{\overset{m}{\underset{j=1}{\sum }}{\left(x_{j}-c_{ij}\right)}^{2}}. \end{array}$$

Above, *x* is the data, *C*_*i*_ is the *i*-th cluster center, and *m* is their dimension. The error analysis and SSE calculation formula for this database are as follows:

(2) $$\begin{array}{c} \text{SSE}=\overset{k}{\underset{i=1}{\sum }}\underset{x\in c_{i}}{\sum }{\left|d\left(x,c_{i}\right)\right|}^{2}. \end{array}$$

In formula (2) ∑_*i*=1_^*k*^∑_*x*∈*c*_*i*__ indicates that the data in SSE can be randomly selected from 1 to *n*, |*d*(*x*, *c*_*i*_)|^2^ indicates that the data objects in the public mental health database extract a cluster center to the SSE for calculation and arrange the calculated SSE values neatly one by one to see if there are obvious wrong data values, if not, put all their values. Add up to determine whether the overall value is changing. If there is a change, it must return to the previous level for reprocessing. If there is no change, proceed to the next step.

Subsequently, we select the optimal data in the public mental health model database for differentiation and increase. At this time, the ID3 algorithm is used for analysis. Extracting and splitting the optimal data in public mental health can help us speed up the analysis of public mental health. The problem of health is that the splitting of data is carried out on the information entropy, and then it is a mathematical formula:

(3) $$\begin{array}{c} \text{Entropy}\left(D\right)=-\overset{m}{\underset{i=1}{\sum }}p_{i}\log_{2}p_{i}. \end{array}$$

If the attribute *a* in the public mental health database is divided, the value of *a* may have

(4) $$\begin{array}{c} V=\left\{a^{1},a^{2},a^{3},\cdots ,a^{v}\right\}. \end{array}$$

By discussing and calculating *a* with formula (3), the information gain of *D* in the public mental health database can be obtained: by discussing and calculating *a* with formula (3), the information gain of *D* in the public mental health database can be obtained:

(5) $$\begin{array}{c} \text{Gain}\left(D,a\right)=\text{Entropy}\left(D\right)-\overset{V}{\underset{V=1}{\sum }}\frac{\left|D^{v}\right|}{D}\text{Entropy}\left({\text{D}}^{V}\right). \end{array}$$

However, information gain likes more useful information value. In order to overcome this shortcoming, the famous C4.5 algorithm is proposed, which uses retrieval speed when selecting attributes, and the calculation formula is as follows. The detailed process of attribute selection is as follows: calculated attribute library. Choose a high level of gain. Then, choose the maximum gain division of these properties:

(6) $$\begin{array}{c} \text{Gain}\_\text{ratio}\left(D,a\right)=\frac{\text{Gain}\left(D,a\right)}{\text{SI}\left(a\right)}. \end{array}$$

In

(7) $$\begin{array}{c} \text{SI}\left(a\right)=-\overset{V}{\underset{v=1}{\sum }}\frac{D^{V}}{D}\log_{2}\frac{\left|D^{V}\right|}{D}, \end{array}$$

the CART algorithm uses the Gini index to select the most appropriate analytical properties and is faster to compute than to compile. The purity of the public mental health database *D* can be measured by the Gini index, and the calculation formula is shown in formula (8):

(8) $$\begin{array}{c} \text{ Gini}\left(D\right)=1‐\overset{n}{\underset{i=1}{\sum }}p_{i}^{2}. \end{array}$$

Equation (8) is expressed as the Gini index, which is used in the model to select the best analytical attribute value in the public mental health database. It is very high, this algorithm is very simple and easy to understand, and it is very consistent with the optimal properties of judgment data.

The concept of the algorithm is very simple, easy to understand, and easy to extract. Target data and digital information can be processed in a way that does not consider information and can handle external features, but also has the disadvantage of being easily overloaded. Second, it is easy to ignore the relationship between features.

### 3.2. Optimizing the Public Mental Health Model

A single decision tree classifier for accuracy and diversity is prone to overload, and unstable classifiers lead to classification problems. Gradient boosted tree algorithms fill these gaps, and the final base classifier is generated to reduce the loss caused by the old base classifier. The loss reduction process includes reducing the residual of the previous weak classifier in the gradient direction and the subsequent accumulation of the weak classifier to obtain a strong classifier. Its basic principles are as follows:

Input: loss function *L* and public mental health model database:

(9) $$\begin{array}{c} T=\left\{\left(x_{1},y_{1}\right),\left(x_{2},y_{2}\right),\cdots ,\left(x_{m},y_{m}\right),\right\}. \end{array}$$

Output: additive model:

(10) $$\begin{array}{c} \overset{\wedge }{f\left(x\right)}=f_{M}\left(x\right). \end{array}$$

The classifier at the beginning:

(11) $$\begin{array}{c} f_{0}\left(x\right)=\arg\min_{\gamma }\overset{N}{\underset{i=1}{\sum }}L\left(y_{i},\gamma \right). \end{array}$$

These classifiers need to perform the following steps:

1. According to *L*, get the negative gradient in each database and use it as an estimated value:

(12) $$\begin{array}{c} r_{im}=-\left[\frac{\partial L\left(y_{1},f\left(x_{i}\right)\right)}{\partial ,f\left(x_{i}\right)}\right]. \end{array}$$

(2) Build a regression tree and get its leaf nodes R_*mj*,_*j* = 1, 2, ⋯, *J*, j. These leaves are quite the type of public mental health
(3) Compute node leaves:

(13) $$\begin{array}{c} {\text{c}}_{mj}=\arg\min_{c}\underset{x_{i\in R_{mj}}}{\sum }L\left(y_{i},f_{m-1}\left(x_{i}+c\right)\right). \end{array}$$

Formula (13) is the function of calculating the leaves of nodes. It plays the role of branches in the system. The whole system is like a tree, and the type of public mental health is the branches and leaves of this big tree. It clearly shows the complexity and diversity of public mental health types, and using the form of leaves as a metaphor for psychological types can be very good for classification and statistics. All leaves on a tree trunk will be of the same type, and the same method can be used. To solve it, the complexity of the system is solved virtually, and the response speed of the system is improved.

(4) Update the regression tree

(14) $$\begin{array}{c} f_{m}\left(x\right)=f_{m-1}\left(x\right)+\overset{J}{\underset{j=1}{\sum }}c_{mjI}\left(x\in R_{mj}\right). \end{array}$$

Output gradient boosting tree:

(15) $$\begin{array}{c} \overset{\wedge }{f\left(x\right)}=f_{m}\left(x\right)+f_{M}\left(x\right). \end{array}$$

The gradient boosting tree algorithm is generated based on the result of the previous tree, which can ensure the continuity of the object. There are many nonlinear transformations, which are very helpful for object transformation and the creation of multidimensional objects. In addition, the slope gradient tree overcomes the tendency of decision trees. It will be excessive, and it is not easy to produce outliers.

### 3.3. Extract Scoring of Data

Filtering evaluates each attribute based on its difference or relevance. And select properties based on preset criteria or selected number of properties. The following are some popular filtering process algorithms, where the variance selection method selects objects based on the difference between each object and its target and the correlation coefficient method, the chi-square test, and the maximum data coefficient law for properties and objectives.

The variance selection method is used to express the degree of deviation of the random variable from the expected value. When using the variance selection method, the variance of each subject is first calculated using the variance formula, and vice versa, according to different needs analysis. Different standard selection rules are defined, and finally, qualified attributes are selected according to the predefined standard selection rules and calculated according to formula (16):

(16) $$\begin{array}{c} s^{2}=\frac{1}{n-1}\overset{n}{\underset{i=1}{\sum }}{\left(x_{i}-\overset{-}{x}\right)}^{2}. \end{array}$$

When using the correlation coefficient method, the correlation coefficient is usually represented by the letter *r*. First, use the correlation coefficient formula to calculate the correlation coefficient for each target geographic feature; second, calculate the *P* value for the correlation coefficient. The *P* value is calculated based on the feature selection target value. The calculation of the correlation coefficient is expressed by formula (17):

(17) $$\begin{array}{c} r\left(X,Y\right)=\frac{\text{Cov}\left(X,Y\right)}{\sqrt{\text{Var}\left[X\right]\text{Var}\left[Y\right]}}. \end{array}$$

The chi-square test is used to find the difference between the actual observed value and the theoretical value. The chi-square is linearly related to the degree of deviation between the actual observed value and the theoretical value. The smaller the chi-square, the smaller the deviation. Hour usually matches the chi-square value of 0 if the actual observed value agrees exactly with the obtained theoretical value. The calculation of the test statistic is shown in formula (18):

(18) $$\begin{array}{c} {ƛ}^{2}=\sum \frac{{\left(f_{a}-f_{e}\right)}^{2}}{f_{e}}, \end{array}$$

where *f*_*a*_ is the observed frequency, and *f*_*e*_ is the expected frequency.

The mutual information method is used to solve the interoperability between two variables. The mathematical formula is

(19) $$\begin{array}{c} I\left(X,Y\right)=\underset{x\in X}{\sum }\underset{y\in Y}{\sum }P\left(x,y\right)\log\frac{p\left(x,y\right)}{p\left(x\right)p\left(y\right)}. \end{array}$$

In L1 regularization, it can calculate the loss of the system, and its function expression is

(20) $$\begin{array}{c} J=J_{0}+\alpha \underset{W}{\sum }W^{2}. \end{array}$$

Among them, *J* represents a function with absolute value, *J*_0_, which is *α* the original loss function, and is a kind of coefficient.

### 3.4. Evaluation Indicators

In order to obtain the public mental health assessment, we use the accuracy rate *T* and the false positive rate *F* as the evaluation indicators for the model we created.

The function expression of the accuracy rate *T* and the false positive rate *F* is as follows:

(21) $$\begin{array}{c} T=\frac{A}{B}\times 100\%, \end{array}$$

(22) $$\begin{array}{c} F_{ij}=\frac{W}{H}\times 100\%. \end{array}$$

Finally, the values obtained by formula (21) and formula (22) are analyzed to summarize the result analysis:

(23) $$\begin{array}{c} Z={\left(T+F_{ij}\right)}^{2}+\ln z_{c}. \end{array}$$

Equation (23) evaluates the entire model. The range of evaluation is very wide. It is the final evaluation function of the system. It combines the previous accuracy rate *T* with the false positive rate *F* and randomly adds a new evaluation factor. This new factor is the opinion of the model, and the purpose of this is to make the model more humanized. If the overall result of *Z* is greater than 1, this indicates that this set of evaluation indicators gives a good evaluation in this model. If the overall result of *Z* is less than 1, then it shows that this set of evaluation indicators gives a bad evaluation in this model.

There are still many areas for improvement in this evaluation system, and we will continue to work hard to improve it in the future.

To analyze the correlation between college music education and public mental health based on deep learning, the public mental health model, clustering algorithm, and filtering algorithm are used. This model has a complete system, which records the information of public mental health into the database. There is also model optimization technology. Even a little error is normal. After all, there are too many factors to be considered in the system. With the continuous development of public mental health, the psychological characteristics and cognitive characteristics generated by this will also be constantly changing and updating, and the system saves these data in each area and solves them slowly.

## 4. Analysis of College Music Education and Public Mental Health in Deep Learning

### 4.1. Deep Learning Analysis of College Music Education

Judging from the current situation of university music teaching, it still maintains a relatively consistent teaching method, which is not conducive to the development of university music teaching nor can it promote the development of music talents. The driving force of social development has entered a new era and must use a variety of abilities to face this situation. Colleges and universities need to expand music education in a diversified direction. At this time, deep learning is introduced to change the university music education model, cultivate versatile university students, and improve the competition in the labor market to enable them to participate in social and economic development. Through the survey, the relevant content of college music education was obtained, and the data are shown in Table 1.

According to the data in Table 1, there are still some unresolved problems in college music education, but the existing education methods can allow students to absorb the knowledge of music education. In response to these problems, my country has increased investment in college education in recent years, using money to invest in it and then adopting the deep learning model to slowly change the status quo of college music education. The following data chart is the amount of investment in recent years and the changes in the direction and direction of college music education reform after investment.

According to the data shown in Figure 1, we can see that my country's investment in college music education is increasing, which shows that my country attaches great importance to the education of music. By 2021, my country's total investment will reach 3.7 billion yuan. Among them, it is the highest. On the contrary, after the decline and rise of classical music, there is basically no change. My country's famous music still needs to be constantly updated. Compared with popular music, it is not very popular among young people.

According to the data in Figures 1 and 2, my country's investment in college music education has increased every year, but this increased amount is not a blind investment but a selective increase in the amount invested in this amount. During the changes, the direction of change in university music education is also different, but in Figure 2, their totality is also rising again. In addition, compared with the previous shallow music learning, there are many benefits of deep music learning.

According to the data in Table 2, it can be known that deep music learning is obviously better than shallow learning. Deep learning can change the attitude of students who do not accept music knowledge and turn them into active learning by themselves. Finally, we specifically investigated a university in our country, hoping to get more useful information from this.

In Figure 3, we can see that both boys and girls have chosen two activities: concert and musical instrument experience class. These are the two most helpful activities for music, and they are the most popular in their universities. Then we investigated them for the purpose of learning music, and we were very satisfied with the final result. Most of them were motivated by interest and wanted to learn music from their hearts.

According to the data in Figures 3 and 4, no less than 55% of the students chose the concert, and nearly 40% of the students chose the musical instrument experience category. While the percentage of lectures and seminars is relatively low, it can be seen from the data in Figure 4 that students often like to listen to concerts, which can also provide a good aesthetic experience, and they are also particularly interested in musical instrument courses. In Figure 5, 90% of the surveyed students choose music class because of their interest. No matter what the reason is, since they choose music class, it shows that they have a certain favorable impression of music.

### 4.2. Public Mental Health Analysis of Deep Learning

Whether the models and algorithms mentioned in experiment 3 are in line with public mental health needs to be further analyzed and explained, and experimental explanations are carried out for many aspects, not only to analyze the mentioned models and algorithms but also to use other to analyze and compare them.

According to the data in Table 3, the public mental model in experiment 3 is generally high in terms of speed and safety performance and is better than other models. Although the data presented by the algorithm is mediocre, however, each has its own characteristics and is sufficient for various operations in the model. There are many problems in public mental health, most of which are listed in Table 4.

According to the data in Table 4, public mental health problems are becoming more and more serious. Anxiety is the most serious problem at present, and the lowest is psychological imbalance. Therefore, we need to solve the problem of people's anxiety and anxiety in a targeted manner, analyze the source of anxiety, and then resolve. For such a serious public mental health problem, we introduce deep learning to optimize and change this phenomenon and discuss and analyze the differences between different household registrations and different genders.

Public mental health has a great influence on people's environment. For example, in Figure 5, it can be clearly seen that there is a big difference in public mental health between people with rural hukou and those with urban hukou, followed by males and females. There are also differences between them. Men's mental health problems are lower than women's. This should be related to the reason why men's psychological pressure is greater than that of women. Finally, after they accept deep learning, their public mental health problems are declining, even in my country of public mental health problems has dropped to a global low, which indirectly illustrates the powerful role deep learning has played in it.

According to the data in Figures 5 and 6, before deep learning was carried out, the public mental health types of the experimental subjects in the two figures were not optimistic. After deep learning, it can be clearly seen from the data that the public mental health level has changed. The psychological endurance of men is stronger than that of women, and people with urban hukou are better than those in rural areas. After deep learning is implemented in my country, the proportion of public mental health personnel in my country has dropped significantly. Our situation has improved markedly in other countries.

From the data in Figure 7, all types in my country are lower than other countries, which also reflects the key role of deep learning in it. At the top is South Korea, whose public psychology health problems are the most serious.

## 5. Conclusion

The theme is the analysis of the correlation between college music education and public mental health based on deep learning, which discusses the definition of deep learning, the difference between deep learning and shallow learning, and the scope of application of deep learning and designs experiments on public mental health model research, which mainly studies the establishment process and optimization system of the public mental health model, extracts and analyzes the system data in a targeted manner, and finally makes a summary evaluation of the entire model. Regarding the problems of university music education and public mental health, we still need to continue to improve. A little research today is not enough to deal with the various problems that will arise in the future. We must continue to study in order to better go forward in the future.

With the continuous changes of university music education and public mental health problems, conventional solutions are no longer sufficient. At this time, we have adopted a method based on deep learning to study them and solve the current situation of university music education. After the frequent occurrence of mental health problems, an in-depth discussion of both of them aims to teach students that they can deeply understand the charm of music and fall in love with music and hope that they can develop in many aspects in their university life. Afterwards, efforts should be made to reduce the proportion of people with public mental health.

## Figures and Tables

**Figure 1:** My country's university music education investment.

**Figure 2:** The trend of university music education reform.

**Figure 3:** Types of activities that a university hopes to increase.

**Figure 4:** The purpose of studying music in a university.

**Figure 5:** Differences in mental health under different household registrations.

**Figure 6:** Changes in mental health by gender.

**Figure 7:** Overall public mental health by country.

**Table 1:** University music education.

Problems with college music education	Features	Teaching methods
Cultivating students' minds	Listen and learn	To enable students to master music knowledge
Exercise learning and creativity	Through sports and games	Improve students' interest in music
Positively influence their worldview	Promote students' self-creation	Deepen students' love of music

**Table 2:** Differences between deep music learning and shallow music learning.

The difference	Deep music learning	Shallow music learning
Music learning attitude	Passive acceptance of learning	Actively learn
Music learning method	Low-end thinking	The operation of high-end thinking
Music learning goals	Basic knowledge and basic skills	Sublimation of thinking, improvement of personal value
Music learning process	Simple, repetitive, and mechanical	Association, transformation, and agility

**Table 3:** Comparison of public mental health algorithms and models.

Compliance	Speed (1-10)	Safety performance
Excellent	8	High
Good	6	Generally
Good	5	Good
Good	7	Good
Good	7	Medium
Qualified	5	Generally

**Table 4:** Overall analysis of mental health.

Good	Mild	Moderate	Severe
1985 (46.6)	1859 (43.6)	374 (8.8)	33 (0.8)
2626 (61.6)	1367 (32.1)	211 (4.9)	43 (0.3)
2860 (67.1)	1081 (25.4)	245 (5.7)	56 (1.3)
2278 (53.4)	1560 (36.6)	358 (3.5)	77 (2.3)
1804 (42.3)	1707 (40.0)	570 (13.4)	14 (1.1)
2181 (51.2)	1749 (41.0)	287 (6.7)	31 (1.8)
3213 (75.4)	930 (21.8)	91 (2.1)	14 (0.5)

## Data Availability

The experimental data used to support the findings of this study are available from the corresponding author upon request.
